The article "Value of CT Radiomics Combined with Clinical Features in the Diagnosis of Allergic Bronchopulmonary Aspergillosis" was published in 2022. Journal: Comput Math Methods Med.

# Value of CT Radiomics Combined with Clinical Features in the Diagnosis of Allergic Bronchopulmonary Aspergillosis

**DOI:** 10.1155/2022/5317509

**Published:** 2022-05-05

**Authors:** Xiaojun Qian, Hengmo Rong, Xue Wei, Guangsheng Rong, Mengxing Yao

**Affiliations:** ^1^Department of Allergy, The Third People's Hospital of Hefei, The Third Clinical College of Hefei of Anhui Medical University, Hefei, China; ^2^Department of Respiratory and Critical Care Medicine, Beijing Chaoyang Hospital, Capital Medical University, Beijing, China; ^3^Department of Respiratory and Critical Care Medicine, The Second Hospital of Anhui Medical University, Anhui, China

## Abstract

**Objective:**

Early diagnosis of allergic bronchopulmonary aspergillosis (ABPA) and targeted treatment can block the process of the disease. This study explores the diagnostic value of CT radiomics combined with clinical features in allergic ABPA.

**Methods:**

A total of 40 patients with ABPA were studied retrospectively, divided into training set (*n* = 28) and test set (*n* = 12). Based on CT imaging, the radiomics features are extracted and combined with clinical features to build a diagnostic model. The diagnosis model was based on support vector machine algorithm. The receiver operating characteristic curve (ROC) and area under the curve (AUC) were used to evaluate the diagnostic efficiency of the model.

**Results:**

There was no significant difference in general information and clinical data between the training and test sets (*P* > 0.05). The AUC of the training set and the test set is 0.896 (95% CI: 0.836-0.963) and 0.886 (95% CI: 0.821-0.952), respectively.

**Conclusion:**

Based on the CT radiomics model combined with clinical data, it has high efficiency in the diagnosis of ABPA.

## 1. Introduction

Allergic bronchopulmonary aspergillosis (ABPA) is an allergic and noninfectious lung disease caused by Aspergillus fumigatus, which is an allergic disease caused by Aspergillus fumigatus [1]. The pathogenesis of ABPA is still unclear, which may be related to genetic factors. After inhaling Aspergillus fumigatus spores, the bronchi of genetically susceptible individuals showed an immune response to Aspergillus fumigatus fungal antigen, which damaged cilia elimination function and acted as a barrier, and caused lung infiltration and proximal bronchiectasis [2]. Due to repeated exposure to Aspergillus antigen caused by persistent fungal colonization in the airway, ABPA is characterized by an early allergic reaction and late lung injury [3–5].

Clinical manifestations of ABPA can be acute or chronic disease courses. The most common symptom is recurrent asthma, and systemic symptoms such as fever, headache, and fatigue may occur during an acute attack [6]. ABPA is not common clinically, and its incidence is low, so it is often misdiagnosed as chronic pneumonia, bronchiectasis with infection, tuberculosis, and lung tumor [7]. Clinically, patients cannot get the correct treatment due to misdiagnosis, and the disease often recurs, eventually leading to pulmonary fibrosis and respiratory failure [8]. Therefore, early diagnosis is of great significance to the prognosis and prognosis of patients.

Radiomics method can transform images into high-dimensional features by machine, and make images digital [9–12]. In recent years, the application of CT imaging omics in medical diagnosis systems has gradually matured [13]. Therefore, this paper aims to explore the diagnostic value of CT radiomics combined with clinical feature diagnosis in ABPA.

## 2. Methods

### 2.1. Clinical Data

A total of 40 patients with ABPA who were clinically diagnosed in the Department of Allergy of The Third People's Hospital of Hefei, Department of Respiratory and Critical Care Medicine of The Second Hospital of Anhui Medical University, and Beijing Chaoyang Hospital of Capital Medical University from 2017 to 2021. There were 16 males and 24 females, aged 21-84 years (50.58 ± 13.77 years). The clinical manifestations are mainly wheezing, cough, expectoration, chest tightness, and history of bronchial asthma.

All the cases were clinically diagnosed, and all of them met the primary and secondary diagnostic criteria of ABPA established by The International Society for Human and Animal Mycology (ISHAM) [14]. Inclusion criteria: (1) bronchial asthma; (2) elevated IgE levels against Aspergillus fumigatus; (3) elevated total IgE levels (>1000 IU/mL); (4) total eosinophil count >500 cells/*μ*L in steroid naïve patients (may be historical); (5) the chest radiographic features consistent with ABPA may be transient (i.e., consolidation, nodules, tram-track opacities, toothpaste/finger-in-glove opacities, and fleeting opacities) or permanent (i.e., parallel line and ring shadows, bronchiectasis, and pleuropulmonary fibrosis). If the patient has symptoms and signs of type I and III allergy and infection of bronchus and lungs by Aspergillus, and Aspergillus hyphae are found on the smear of deep bronchial secretion or Aspergillus grows for many times, it can be diagnosed as ABPA [15]. Exclusion criteria: (1) the patient already has severe pulmonary dysfunction and (2) possible lung malignancies. In this study, 40 patients met the above diagnostic criteria.

### 2.2. Instruments and Methods

GE64-row light speed spiral CT was used to scan, and all graphic raw data were transmitted to the ADW4.4 workstation for postprocessing. Scanning parameters: tube voltage 140 kV, tube current 300 mA, rotating speed 0.6 r/s, screw pitch 0.984: 1, collimator width 0.625 mm × 64 layers, and scanning layer thickness 0.625 mm. The lung window was reconstructed by the bone algorithm, and the thickness of the reconstructed layer was 1.25 mm. The mediastinal window was reconstructed by the soft tissue algorithm, with a reconstruction layer thickness of 5 mm, a reconstruction interval of 0 mm, and a matrix of 512 × 512. All patients were in a supine position with their hands on their heads, and the scanning range was 3 cm from the thoracic entrance to the diaphragm. Enhanced chest scan: use nonionic iodine contrast agent with a concentration of 320 mgI/ml, dosage of 1.3 ml/kg, and the scanning parameters are the same as those of plain scan.

### 2.3. Image Segmentation

At the level of the most significant section of the image lesion, the image window width and window position is unified (set the window width of 400 Hu and the window position of 40 Hu). Then, using ITK-SNAP 3.8 software, the regions of interest (ROI) are delineated along the lesion contour. An attending physician with 10 years of working experience in radiation diagnosis specialty used the blind method to check the outlined ROI (Figure 1). Import the maximum slice image of the focus-enhanced CT horizontal axis, and the corresponding ROI image was drawn into A.K. software for feature extraction. There are 396 features extracted from the axial images of the largest slice of each lesion, including morphological features, first-order histogram features, second-order histogram features, and higher-order features.

### 2.4. Feature Extraction

Patients were randomly divided into training group (*n* = 28) and verification group (*n* = 12) according to 7: 3. First, standardize the data indicators to eliminate the influence of the difference between dimensions and value range. The minimum redundancy maximum correlation (mRMR) algorithm is used to preliminarily screen the features in the training set, eliminating redundant and irrelevant features and retaining the features with the greatest prediction efficiency.

(1) $$\begin{array}{c} \text{mRMR}=\begin{array}{c} \text{argmax}\\ f_{i}\in X \end{array}\left[I\left(c;f_{i}\right)-\frac{1}{\left|S\right|}\underset{f_{j}\in S}{\sum }I\left(f_{i};f_{j}\right)\right]. \end{array}$$

In this study, the “minimum-maximum normalization” is used to linearly transform the original data and map the data to [0, 1], to facilitate comprehensive analysis and make the results more accurate.

(2) $$\begin{array}{c} \text{NMIFS}=\begin{array}{c} \text{argmax}\\ f_{i}\in X \end{array}\left[I\left(f_{i};c\right)-\frac{1}{\left|S\right|}\underset{f_{j}\in S}{\sum }\frac{I\left(f_{i};f_{j}\right)}{\min\left(H\left(f_{i}\right),H\left(f_{j}\right)\right)}\right]. \end{array}$$

Finally, the least absolute shrinkage and selection operator (LASSO) algorithm is applied to further screen the remaining omics features. The objective function of the prediction model based on LASSO regression is expressed as follows:

(3) $$\begin{array}{c} \overset{n}{\underset{i=1}{\sum }}{\left(y_{i}-\overset{p}{\underset{j=1}{\sum }}x_{ij}\beta_{j}\right)}^{2}+\lambda \overset{p}{\underset{j=1}{\sum }}\left|\beta_{j}\right|=\text{RSS}+\lambda \overset{p}{\underset{j=1}{\sum }}\left|\beta_{j}\right|. \end{array}$$

### 2.5. Establishment and Verification of the Model

A support vector machine (SVM) classifier is used to build a diagnosis model by combining clinical factors and imaging characteristics. The linear inseparable data of SVM is projected into the high-dimensional space by mapping function, so that the features become linearly separable in this space, and then the features are divided by a hyperplane with the maximum boundary interval. The effectiveness of training set and test set models is verified. The specific process is shown in Figure 2.

## 3. Result

### 3.1. General Information and Clinical Data

General information and clinical data of patients in the training set and the test set were analyzed. There was no significant difference in gender, age, wheezing, cough and expectoration, fever, wet sound, wheezing sound, total IgE, and aspergillus between the training set and the test set (*P* > 0.05) (Figure 3).

### 3.2. Selection of Image Features

A total of 936 radiomics features were extracted, and 6 optimal radiomics features were obtained after processing, namely, the squareroot-glcm-inverse variance (Squareroot-IV), the square-glcm-inverse variance (Square-IV), the exponential-MCC (E-MCC), the squareroot-MCC (S-MCC), the firstorder-kurtosis (FK), and the small dependence low gray-level emphasis (SDLGLE).  Figure 4 shows the six imaging features arranged according to the weight coefficient from low to high.

### 3.3. Composition and Prediction Efficiency of the Model

The diagnosis model consists of the clinical data of central bronchiectasis; mucoid impaction of dilated bronchial, a cylindrical capsule like toothpaste; patchy infiltration; and centrilobular nodules with a tree-in-bud pattern, and extracted six radiomics characteristics. In the training set, the area under the curve (AUC) of the model was 0.896 (95% CI: 0.836-0.963). In the test set, the AUC of the model was 0.886 (95% CI: 0.821-0.952). The diagnosis model has high prediction efficiency (Figure 5).

## 4. Discussion

ABPA is mainly caused by Aspergillus infection, and Aspergillus fumigatus is the most common clinically. Healthy people rarely cause ABPA because of the function of the bronchial mucosa-epithelial barrier, mucociliary clearance, and phagocytosis of alveolar macrophages. ABPA is common in patients with asthma or cystic fibrosis, and it is also related to the gene-phenotype of the host [16]. When Aspergillus is inhaled by genetically susceptible individuals, it releases antigens, proteolytic enzymes, and other toxic substances activate T lymphocytes, releases interleukin- (IL-) 4, IL-5, and IL-13, and secretes IgE and IgG antibodies, which act on mast cells, alveolar macrophages, and eosinophils, causing an inflammatory reaction in the airway wall and surrounding lung tissues, leading to increased secretion of mucus glands accompanied by bronchospasm [17, 18]. With the development of the disease, bronchial mucus impaction and eosinophil pneumonia can be seen, followed by bronchiolitis obliterans and pulmonary interstitial fibrosis [19].

ABPA can occur at any age, but most are middle-aged and older adults, and there is no obvious gender difference [20]. Clinical manifestations can be acute or chronic disease course, the most common symptom is recurrent asthma, and systemic symptoms such as fever, headache, and fatigue may occur during acute attack [6]. HRCT examination showed central bronchial and pulmonary parenchyma changes, and blood examination showed eosinophils in peripheral blood increased. Immunological examination showed serum total IgE, Aspergillus fumigatus IgE, and IgG antibody increased [21]. Our study shows that IgE and eosinophils in ABPA patients are significantly increased. Muthu et al. [22] systematically evaluated and meta-analyzed previous studies. Their results showed that recombinant Aspergillus fumigatus antigen-specific IgE might play an essential role in the early diagnosis of ABPA.

Pathological features of ABPA mainly include central bronchiectasis and noncaseous granuloma formation [23]. The main change is central granuloma in bronchi and bronchioles, which is characterized by edema of the bronchial wall and infiltration of inflammatory cells such as eosinophils. Central bronchiectasis is dilated affected segment, subsegmental bronchi, and normal distal bronchi. Soft tissue density mucus plugs can be seen in the lumen of dilated bronchi. The main components of mucus plugs are mucus and Aspergillus filaments [24]. If the disease worsens repeatedly, the airway structure will be destroyed permanently, eventually leading to pulmonary interstitial fibrosis [25]. Central bronchiectasis; mucoid impaction of dilated bronchial, a cylindrical capsule like toothpaste; patchy infiltration; and centrilobular nodules with a tree-in-bud pattern may appear on chest CT in patients with ABPA, but pleural effusion is rare on imaging [26]. Patients with ABPA with central bronchiectasis and high attenuation mucus embolism are the most serious and prone to repeated attacks. Therefore, an early and effective diagnosis is crucial for the individualized treatment and prognosis of ABPA.

The clinical diagnosis of ABPA is mainly based on the following clinical indicators: whether there are asthma symptoms, the rapid positive reaction of Aspergillus antigen skin test, a noticeable increase of serum IgE and IgG antibody titers, and the diagnosis is made in combination with imaging data [27]. In this study, the diagnostic efficacy of ABPA was evaluated by constructing CT radiomics combined with clinical data. In this study, 6 imaging omics features were included in the prediction, and the AUC in the training group, and the verification group reached 0.896 and 0.886, respectively, showing good diagnostic ability. This result is similar to previous studies [28]. Radiomics is to transform cross-sectional image arrays (such as CT, MRI, and PET-CT) into quantitative image features. Essentially, it is to digitize images for accurate quantitative analysis [29–31]. A large number of image data can realize the integration of medical data that cannot be achieved by conventional imaging. Compared with the traditional morphological diagnosis mode, it is more detailed, objective, and accurate, which may be the reason for the higher diagnostic efficiency of radiomics model [32].

## 5. Conclusion

There is a correlation between the CT radiomics model and some imaging characteristics of ABPA. Based on clinical data, the radiomics characteristics are expected to become a new means of diagnosing ABPA. There are several limitations to this study. First, the sample size is small. Second, the ROI of lesions is manually segmented by radiologists, which is influenced by the subjective consciousness of observers to some extent. In addition, this study is retrospective, and there is some bias.

## Figures and Tables

**Figure 1:** Delineation of lesion region of interest. (a) Bronchial showed “tree-in-bud sign”. (b) Magnification of region of interest.

**Figure 2:** The process of model establishment and verification.

**Figure 3:** Comparison of patient information and clinical data between training set and test set.

**Figure 4:** Optimal tuning parameter screening, feature dimensionality reduction, and optimal feature importance ranking chart.

**Figure 5:** ROC of training set and test set models. (a) Training set; (b) test set.

## Data Availability

The data used to support the findings of this study are available from the corresponding author upon request.
